# Analysis of Agriculture and Food Supply Chain through Blockchain and IoT with Light Weight Cluster Head

**DOI:** 10.1155/2022/1296993

**Published:** 2022-08-10

**Authors:** Anass Hamadelneel Adow, Mahendra Kumar Shrivas, Hussain Falih Mahdi, Musaddak Maher Abdul Zahra, Devvret Verma, Nitika Vats Doohan, Asadullah Jalali

**Affiliations:** ^1^Department of Accounting, College of Business Administration, Prince Sattam Bin Abdulaziz University, Al-Kharj, Saudi Arabia; ^2^Department of Computer Science and Engineering, O. P. Jindal University, Raigarh, India; ^3^Computer Engineering Department, College of Engineering, University of Diyala, Baqubah 32001, Iraq; ^4^Computer Techniques Engineering Department, Al-Mustaqbal University College, Hillah 51001, Iraq; ^5^Electrical Engineering Department, College of Engineering, University of Babylon, Hilla, Babil, Iraq; ^6^Department of Biotechnology, Graphic Era Deemed to be University, Dehradun, Uttarakhand 248002, India; ^7^Department of Computer Science and Engineering, Medi-Caps University, Indore, India; ^8^American University of Afghanistan, STM (Science Technology Mathematics), Kabul, Afghanistan

## Abstract

By 2050, the world's population will have increased by 34%, to more than 9 billion people, needing a 70% increase in food production. Prepare more dishes with fewer ingredients. Therefore, the critical goal of manufacturers is to increase production while being ecologically benign. Supply chain systems that do not enable direct farmer-to-consumer connection and rising input costs influence data collection, security, and sharing. Constraints on data security, manipulation, and single-point failure are unfulfilled due to a lack of centralized IoT agricultural infrastructure. To address these issues, the article proposes a blockchain-based IoT model. This study also shows one-of-a-kind energy savings. The decentralization of data storage improves the supply chain's transparency and quality through blockchain technology, thus farmers can engage more efficiently. Blockchain technology improves supply chain traceability and security. This article provides a transparent, decentralized blockchain tracking solution and proposes an intelligent model protocol for several Internet of Things (IoT) devices that monitor crop development and the agricultural environment. A new approach has resolved the bulk of the supply chain difficulties. Smart contracts were utilized to organize all transactions in decentralized supply networks. The use of blockchain technology improves transaction quality, and customers may verify the legitimacy of an item's authenticity and legality by using the system. A total of 100 IoT nodes were distributed randomly to each 500 m^2^ cluster farm. The Internet of Things nodes were used to assess soil moisture, temperature, and crop disease. Network stability period and network life of the proposed method show 90.4% accuracy. The food supply chain will be more efficient and trustworthy with an intelligent model. The immutability of ledger technology and smart contract support further increases supply chain security, privacy, transparency, and trust among all stakeholders in the multi-party system. By 2050, the world's population will need a 70% increase in food production. The food supply chain will be more efficient and trustworthy with an intelligent model. This article provides a transparent, decentralized, and intelligent model protocol for several Internet of Things (IoT) devices.

## 1. Introduction

According to the United Nations Population Division, there will be 10.9 billion people by 2050 [1]. Food production must rise in lockstep with global population growth, also natural resources should be protected. Remember that food and agricultural markets are vital for long-term prosperity [2]. Modern agriculture presents several environmental and social challenges. Farmers have limited control over necessary natural resources such as land and water. Dietary and consumer habits, as well as weather changes, all impede food delivery. Current agricultural practices cannot produce sustainable food and agriculture due to deforestation, water shortages, and soil erosion. Modern and more efficient technologies must be used to preserve resources while boosting productivity. Smart farming is akin to adapting to “holistic” practices [3]. Smart agriculture is a climate-change-aware approach to agricultural land management. A group of colleagues developed the notion of smart agriculture in 2009, arguments about climate change and sustainable development have given rise to smart agriculture [4]. Smart agriculture both combats global warming and ensures food security.  Figure 1 depicts the data-driven farm management cycle, in which crop information is processed using sensors and then sent to a platform where the data is analyzed using the software. After looking at the input, artificial intelligence (AI) turns it into a decision that can be used by acting on it.

### 1.1. Internet of Things in Smart Farming

IoT in agriculture monitors soil, plants, livestock, and the environment. The IoT is used in an IoT-enabled smart farm. Farmers' output has increased, therefore. The biomass of soil and plants is being evaluated. IoT-based sensors can also be used to monitor soil moisture and pests along with crop progress and yields. Farmers may also employ crop rotation to adapt to changing circumstances [5]. Agri-IoT applications aid in agricultural planting and irrigation. In-vehicle Internet of Things sensors for livestock, transportation, and agriculture has the potential to improve [6]. It shows how cattle, land, and crops are processed and the result.  Figure 2 also shows the food and agricultural supply chain process [7].

Constraining risks, delays, and disruptions may be challenging at times. One such solution is blockchain [7, 8]. One that protects and anonymizes data. Only the owner should transact if data is distributed. Other network devices should also be double-checked. It shields inter-node transactions [9]. It is often controlled by the owner or a trusted intermediary (such as a bank). In a typical centralized computer system, everything is controlled by a single server [10]. Each block contains hashes of the previous and the current blocks.

A sender node initiates a transaction, and validation occurs at receiving nodes. It is the node that successfully completes the proof of work. The sender must additionally provide the recipient's public key. Therefore, the transaction may be verified by any node. Each block carries the hash of the block before it. Transactions can be broadcasted and relayed in a variety of ways, all of which are decided by the nodes and miners involved. The network's miners are in charge of verifying transactions by merging batches of transactions into blocks and then delivering those blocks farther into the network. Nodes are responsible for receiving these blocks and then distributing them after confirming that miners respect the network's regulations. Blockchain technology might be the next step toward more openness and accountability in the food supply chain shown in Figure 2. Food products will be visible throughout the supply chain. Using blockchain and IoT, monitoring and sensing food items in real-time reveals supply chain bottlenecks. Pesticides are often sprayed on plants before harvesting, putting customers' health at risk. There is also food fraud and computer hacking.

### 1.2. Blockchain and the Food Chain

This computerized database manages and tracks digital and physical resources. The use of blockchain technology improves transaction quality [11–14]. Customers may utilize the blockchain to verify an item's authenticity and legality.  Figure 3 depicts how blockchain may relate to the food chain; the ability to track the path of a product aids in regulation and legal accountability. Regardless of the manner of transmission, smart contracts play a critical role in this scenario. When the supply chain goes from the end-users to the merchants, it is then controlled by a blockchain-based supply chain system with certifiers from well-known groups.

This link is recorded in blockchain [15], the Internet of Things (IoT) and blockchain are vital components of the digital revolution. The amount of data and connected devices on the Internet of Things will grow. As a result, we have the IoT. 2.0 getting helpful information from IoT devices and data. If IoT efficiency increases by 2030, blockchain is expected to produce $176 billion [16].

### 1.3. Blockchain and IoT Assumptions in 2030

A lack of total food traceability today causes health and food safety risks, hunger is the leading cause of death around the globe [17]. On the other hand, IoT with blockchain will eliminate the need for any third party and create a decentralized system. Customers are worried about the quality of the food they purchase. It is difficult to attract clients in a limited location. IoT and blockchain can increase customer trust. This architecture ensures that data is sent from the maker to the retailer [18]. Connected IoT and apps norms, protocols make network communication easier. Because of the Internet of Things' protocols, both low- and high-power devices can connect to it. The protocols used by the Internet of Things enable devices connected to the network to communicate and share data. HTTP, LoRaWAN, Bluetooth, and Zigbee are just a few protocols that are often utilized in IoT applications. LoRaWAN is a wireless network that connects sensor nodes to the cloud. Scalability and flexibility were desired to communicate with other IoT devices and offer new services [19]. Heizelmann developed the low-energy adaptive clustering hierarchy (LEACH) method. Each protocol node has its own administrator. Sensor data from member nodes is sent to the base station through CHs. Smart agriculture may not only meet crops' fundamental requirements, but it may also forecast their individual needs while taking environmental factors into account. Crop losses might be challenging to predict. Farmers may use IoT nodes to collect and exchange data [20].

### 1.4. Agriculture and the Internet of Things

Soil, water, and field conditions would be monitored remotely, the method assists farmers in making choices that will increase agricultural productivity and efficiency. Farmers may be able to boost agricultural output by using IoT networks and a user-specific web application [21]. An Internet-of-Things-enabled agricultural data processing system to transfer data from the field to farmers using a web application was employed. Moisture sensors in the soil and ultrasonic sensors technologies are low-cost yet high-energy. The authors used IoT to help Indian farmers, farmer suicides have occurred in India because of poor agricultural production. Our smart farm system employs IoT to monitor pests and soil moisture. Agribusinesses' improved seeds and increased harvests, the system is robust, but it is expensive. Innovating and adapting to climate change will help farmers reduce their carbon impact. Research articles were published between 2016 and 2018, covering sophisticated IoT farm applications and sensor data. Smart agriculture manages water, grain, animals, and irrigation, these simulations accumulated the most sensor data.

## 2. Literature Review

This section examines blockchain research in agriculture, blockchain technology is gaining traction in agriculture, banking, finance, and intelligent and transparent governance. Based on risk analysis and critical control points, a blockchain and IoT-based agricultural food supply chain traceability approach was proposed [22]. Hyperledger and Ethereum are being used to track a product from the producer to the customer. In [23], they also put food traceability in place and expressed concerns regarding food safety and security. Agri-ICT in blockchain was investigated and improved, accordingly [24] proposes “smart contracts and DLT efficiency.” There are hazards and challenges in using blockchain in the food supply chain, [25] proposed an IPBFT-based blockchain system for food supply chain buyers. Grain quality is being monitored via blockchain smart contracts. When you utilise a blockchain, you can track every stage of a product's life cycle, from the moment it is developed to the moment it is acquired by a client. DNA from farm animals and pesticide residues, for example, may be preserved in a secure and safe setting while being unaltered. Any company participating in the product's distribution chain can investigate and confirm this information. The expense of gathering data for everything may be prohibitively expensive, but sampling may be used instead. The study investigated how blockchain-based technologies may benefit small-scale farmers [26]. The authors proposed [27] blockchain to improve transparency and process automation in agriculture, [28] presented a blockchain traceability system based on Hyperledger. According to the linked study, blockchain technology increases data security, transparency, and verification. Analysis by the cryptocurrency chain researchers showcased rapid trust development in disaster relief supply networks as a theoretical model [29]. Collaboration reduces lead times and increases supply chain transparency, enhancing supply chain resilience by removing knowledge asymmetry. Incorrect data may undermine a company's reputation. They advocate the use of blockchain technology to increase “trust” among supply chain participants. This solution consolidates all processes in a hypothetical supply chain arrangement into a single database. The database is in charge. This method has drawbacks. The server manages the database. As a result, if one server fails, the whole system fails. Data may be updated without the stakeholders' knowledge [30]. Such ruses are prohibited, we, too, are enigmatic. Product traceability, stakeholder transparency, and trust are key difficulties in the supply chain ecosystem. An overabundance of intermediaries erodes confidence and performance [31].

Farmers', wholesalers', and retailers' food-related outbreaks will be challenging to track. It is also relatively centralized, various groups lack trust in one another, and traceability is essential. Trust concerns in the supply chain may cost businesses much money, companies work hard to gain the confidence of their customers. Access to data while restricting unauthorized changes should be beneficial. These risks may be alleviated by new supply chain technology, and blockchain technology has the potential to improve supply chain efficiency and solve inefficiencies. Blockchain also addresses supply chain issues by using distributed ledger technology. Its impermanence and scattered nature give security, transparency, and new technology may help ecosystems [24].

There is a lack of traceability, visibility, and efficiency in agricultural and food supply networks [32]. Blockchain improves food safety and quality while decreasing supply chain costs. When a product's demand unexpectedly increases, a typical supply chain must be developed. Customers may benefit from supply chain management as a computerized system records the flow of commodities and information depicted in Figure 1 with various stakeholders such as farmers, suppliers, manufacturers, distributors, and retailers. Data loss, manipulation, and security concerns are common in conventional centralized supply chains. Transparency is a typical supply chain issue.

1. There is no information about the origin.
2. There is no assurance of food safety.
3. There are no transaction records in the supply chain.

Blockchain technology acts as a public ledger across networks, addressing difficulties such as verification and validation. Blockchain technology assures security, eliminates intermediaries, lowers transaction costs, and increases product quality. The use of encryption here boosts user confidence and, as a result, product demand [29]. Therefore, each blockchain block includes transaction data, the chain adds a new genesis block. A hash value connects each block, blockchain is a new technology that has the potential to revolutionize several areas of collaboration. Peer-to-peer networks are linked directly with each other and keep their own copy of the distributed ledger. Its characteristics promote trust and openness in collaborative environments. A single political party or organization does not govern it, this feature enables transaction tracing. It is responsible for refreshing the distributed ledger and making it available to all nodes. As a result, it is hard to cope with the distributed ledger, unlike traditional databases, which cannot be modified or erased. Consider blockchain-based smart contracts, computer programs define formalized paraphrase contract logic.

When preliminary data is sought, the “search for origin” may assist in resolving business difficulties. A blockchain-based system can monitor the sources of transactions. Transactions may be tracked all the way back to their inception, when acquiring, a company looks for a mediator. Tracking exact quantities across partnership firms or subsidiaries has historically proved challenging. The blockchain has the potential to automate this process, almost all transactions are now conducted on the blockchain. With distributed ledgers, order tracking is feasible auditors are often hired only for the purpose of the job [33]. By eliminating human interaction, blockchain simplifies and speeds up audits.

Then, grant extra permission, the attackers are unable to alter the transactions. Once recorded, immutable blockchain transactions cannot be modified or reversed. Nobody, not even the administrator, has the authority to reverse previous transactions. Because blockchain technology employs the hash function, changing the data also gives a different hash. All blockchain nodes share a decentralized ledger, these are recorded in the ledger of each node. Those who pursue self-gratification will fail, every transaction on the blockchain must be approved unanimously.

While blockchain removes intermediaries, smart contracts are required to bind contributions and limit distrust. Smart contracts, like conventional contracts, provide organizational norms and conditions for maintaining trust. A controlled code carries out the agreement's regulations, terms, and conditions. Since the 1980s, an intermediary-free smart contract has existed. Nick Szabo [34] came up with the idea. A smart contract encrypts contractual commitments, making them more difficult to breach. As a result, smart contracts limit attacks, the Ethereum network popularised smart contracts and their use in 2016. Smart contracts and integration options are available on the blockchain platform. Smart contracts automate blockchain operations, in various cases, decentralized applications (DApps) store contracts and are used to implement business contracts. Automation makes real-time product tracking and process visibility possible, adding the necessary functions, modifiers, and events to a smart contract. Contract encryption inside the blockchain may allow parties to trust one another.

CAIPY is an IoT-based car insurance ecosystem that uses tamper-proof IoT sensors to monitor a vehicle's state [35]. Smart contracts may be used to manage intellectual property rights. BMC protector is a blockchain-based network for music copyright. From music creation to royalties' distribution, their smart contracts encompass it all. Because smart contracts are immutable, they must be used within a blockchain ecosystem to ensure maximum security. Smart contracts often employ attributes, functions, events, and modifiers. A memory variable with a value is referred to as an attribute, integers, strings, doubles, mappings, addresses, and enumerators are all supported by Solidity. In a system, functions are defined by procedures and responsibilities. When a function is called, it performs its function.

## 3. The Proposed Model for IoT

Enabled smart agriculture has received more interest than blockchain-enabled food supply systems. Most solutions are fictitious. We developed an intelligent future model that employs IoT and blockchain to enable traceability across the food supply chain, thus meeting the demands of all stakeholders. Therefore, we need a distributed, efficient, and secure system for product monitoring and food fraud prevention. The goal is to automate agricultural food supply chain traceability to meet changing consumer expectations. End-to-end data security is provided through smart contracts and transaction data.

### 3.1. Protocol for Smart Models

This section defines the smart model protocol for several Internet of Things (IoT) devices that monitor crop development and the agricultural environment shown in Figure 4. A GPRS router is used for wireless telemetry, and the RFG gateway connects two data streams, enabling cluster farm equipment to be remotely viewed and operated. The SQL database server's logical data layer is where data is stored. Because of a SQL query, the SQL database is accessed for raw data.

The primary goal of the research is to save energy since every network requires it. These include nodes, cluster heads, and sinks. IoT nodes transmit data to CH, subsequently distributing it to sinks to relay data to the base station. An RFG server was built using a TS7260 single board chip (SBC) in this project (SBC TS7260). The system switches modes, the SBC sleep mode is powered by the UPS, and the bulk of cluster farm devices utilizes RS232 serial. Wireless routers are switched off to save battery power while the system is asleep. The SQL server collects data by pulling or pushing it, which allows the server to react quickly to new data. SQL discovers the data, and the data manager can recover and resend lost data packets. Each new data source requires minor modifications to the database and web display layer. Codes are used to connect nodes and observations.

### 3.2. Intelligent Blockchain Modeling

Food safety will be improved by merging agricultural and food supply chain activities, Figure 5 shows how the blockchain works. Stakeholders in the system are also addressed, and data was sent between blockchain mining nodes. AI control monitors and violation notifications may be shared between parties, smart contracts are used to identify food supply chain theft. Speed, size, and automation are the three aspects of AI that have contributed to its use in the first place for the purpose of information gathering. In terms of the speed of computation, artificial intelligence is already quicker than human analysts, and this advantage may be further improved by the incorporation of new technology. Actually, artificial intelligence is the only technology that can analyze enormous volumes of data in an acceptable period of time. This is due to the inherent qualities that AI possesses in this domain. Lastly, but certainly not the least, an algorithm for machine learning may function on its own, which would make the process of analysis more time and labor effective.

Seed dealers organize and create seeds to sell to farmers, high-quality seeds are required for a successful harvest. Thanks to the blockchain, everyone may now exchange data on seed germination and chemical composition. The serialized Global Trade Identification Number is used to monitor and identify seeds. When a farmer purchases and plants high-quality seeds, the farmer must keep the MPEG files, including data from planting through harvesting on several nodes. On the other hand, farmers may utilize the blockchain to directly communicate with clients and sell their produce, avoiding the necessity of intermediaries.

Crop buyers purchase and sell unprocessed crops, the grain is bought and inspected for moisture levels by the processor. Other supply chain participants may access data recorded on the processor's blockchain, blockchain technology has the potential to significantly assist the agriculture industry. The use of blockchain technology in agriculture can lead to improved trust among stakeholders, more efficient information sharing, and cheaper transaction costs. Agro-storage—agricultural storage is inextricably tied to agricultural production and supply chain activities. Grain is stored on the blockchain for supply chain parties to view and trade.

Producers and distributors work together, many distributors have exclusive purchase contracts restricting their market access, while the distributor is the only point of contact for potential customers. Distributors, on the other hand, seldom sell directly to retailers, wholesalers will purchase large quantities of an item that the distributor or manufacturer does not have in stock. All product data must be stored on the blockchain, retailers profit from direct customer sales. Shopkeepers explore the market for bargains and acquire a modest quantity from a distributor. Buying in bulk with traceable IDs simplifies product life cycle and data analysis.

Customers may follow the manufacturing process from beginning to end, participants must digitally sign the transactions and execute the smart contracts, further recorded in the blockchain through the consensus process. All participants give correct data to avoid penalization, and the systems collect pictures automatically and store them on the blockchain for audits. Product traceability helps all parties in the food supply chain, WSN nodes use more energy and cluster less successfully than IoT nodes. This study resulted in developing a unique LEACH-based clustering method for IoT-based agriculture.

Mechanisms of clumping cluster farms are made up of groups of IoT nodes, each with its own head node.

1. CH amplification: alternative CH amplification is required before sending data to the base station. The CH selection method considers node history as well as optimal node proportion. Nodes are picked at random (between 0 and 1), and the node is CH if Tn is chosen at random.
2. Information flow: turn off the member node before transmitting data to save energy. The CH must keep the receiver turned on and merge all the data into a single signal to send an entire message.
3. Navigation: the selection of traffic routes is referred to as “routing.” Farmers may utilize the agricultural IoT network data to analyze and make decisions. There are three data-routing levels in it: member, CH, and sink. The sink saves CH energy while minimizing packet losses.
4. Configuration: the first round uses an equation to produce LEACH CHs and pick cluster heads. Each network node expends energy to transfer, send, and receive data. Because all nodes in a cluster farm begin with the same amount of power, the sink node may be located wherever. The intensity of the node signal influences first-round placement, during this technique, GH stops detecting data. There is much energy leftover in the cluster heads at the sink and GH. This distance is calculated separately for each dimension. Because the total number of cluster heads has decreased, certain cluster members will find it more difficult to communicate with their individual cluster leaders. The frequent connection between cluster heads will raise the amount of energy consumed and lower the network's lifespan if there are too many cluster heads. The BS's power requirements are significantly more specialised than those of standard operations. In contrast to the usual LEACH approach, the threshold value strategy selects CH at random from a set of energy-dependent attributes.

The energy consumption of a node is affected by network density, packet size, and network density. EL and TL have an inverse relationship. A low TL indicates a high EL, notify all nodes if the EL settings do not minimize the remaining energy. Only data-transfer nodes remain active to save energy. The base station saves bandwidth by integrating data from all sensing member nodes into a single hop. Because blockchains are not managed by a single body, they may operate without a hitch. An administrator is the only person who can control and own all of the data stored within a database. Despite their classification as two distinct technologies, databases and blockchains may be merged into a single operating system provided the proper steps are followed.  Figure 6 depicts the IoT-based agriculture cluster farm and data transmission.

### 3.3. Concurrent Assumptions

Before death, the node is calculated using ideal values that vary with node density. A total of 100 IoT nodes were distributed randomly to each 500 m^2^ cluster farm. The sensor nodes that will be used to monitor the environment are intended to be installed in the field and linked to the centralised application through CH nodes. The CH is in charge of data gathering and processing, as well as forwarding processed data to the BS for further investigation. Data collected from all the sensors will be relayed to the BS through the CHs at the start of each round. The Internet of Things nodes were used to assess soil moisture, temperature, and crop disease. Cluster nodes are scattered such that they can only communicate with cluster leaders in their own cluster. The sink node talks with the BS on the CH's behalf, and a little message is sent across a great distance using the widely utilized LEACH.  Figure 7 depicts a comparison graph of the old IoT-based model and the suggested model with several rounds vs stability period and rounds vs energy consumption, demonstrating the proposed method's superior performance. In the proposed model with a good SNR, the first-order radio model sending an *m*-bit message across *d* distances should result in fewer I/O losses than using the radio model. As a result, protocols have to cut down on how far messages have to travel and how long it takes to send and receive each one.

### 3.4. Modifiers Improve Actors or Components

Editing or access rights may be granted to other actors or components. A blockchain transaction log records information about an incident. Any event parameter is recorded in the transaction logs of the blockchain. This strategy allows the recovery of system history in the future. Smart contracts are blockchain-enabled computer programs. A contract is usually automated to reduce the need for intermediaries and wastage time. Contracts created in the blockhain are inefficient. It is difficult to track and document evidence in the traditional supply chain since it is paper-based or multiple parties maintain their own systems, which are not accessible to each other. When specific circumstances are satisfied, smart contracts are executed quickly, removing the need for a mediator. This kind of code-based contract enables quick action execution (like payments). It differentiates the blockchain from Ethereum, a smart contract pays the transporter when a client verifies a shipment.

A smart agreement between two parties, for example, ensures that the arrangement is carried out, unlike a traditional contract. Parties may engage more simply and transparently using smart contracts, smart contracts may be found at their own addresses. This address is never used to modify blockchain records, instead, it holds the smart contract code in the blockchain platform. All consensus nodes participate in the transaction. Smart contracts may be either deterministic or non-deterministic in nature. A deterministic smart contract operates without the involvement of a third party, this is a smart contract that is non-deterministic (database). A smart contract's blockchain code comprises “if/when...” lines.

When certain conditions are met, a computer network will act, and the transaction is then recorded on a blockchain. Unless otherwise indicated, only authorized parties may investigate the ramifications of a transaction. Blockchain technology should assist supply chain managers in resolving coordination issues. Smart contracts may be used by many parties, lowering complexity, boosting supply chain transparency, and improving trust-free verification. If blockchain technology is used to execute the system, global supply chains may be able to work without the involvement of third parties. Furthermore, it promotes greater integration of financial and logistical services, as well as an improvement in data communication across a wide range of stakeholders. The supply chain will also be made simpler and more adaptable. Combining blockchain with smart contracts results in an automated, secure, and innovative solution. Smart contracts handle business logic and data access.

### 3.5. Model Outcomes Proposed

After collecting sufficient data, we constructed our conceptual model, which incorporates parts of the current manual and blockchain-based agri-food supply chains. Farmers get seeds from suppliers. In addition to the information on the seeds, seed suppliers, and harvests, we provided the network with a complete document. The blockchain will be used to store transactions after analyzing his seeds and crops, a farmer places an on-the-spot order. The unprocessed rice is fed into the processor, the distributor oversees the contract once the processor gets it. The shop's purchase order comes next, the distributor then sends orders to the merchant after uploading a shipping document. Wholesalers provide wholesale rice to retailers for retail sale to consumers. The buyer has complete access to the history of the rice, from harvest through the sale. Smart contracts enable two parties to interact with one another.

Consensus lends validity to this concept; consensus governs transaction validation. The validator node, for example, will alert the data source, it will be notified after the transaction is completed. They provide permission for legitimate transactions; a validator may reject an invalid transaction. This article suggests a permissioned blockchain system based on Ethereum, it is a completely decentralized architecture that employs cutting-edge technologies such as blockchain to guarantee proper supply chain operation. We have theoretically researched smart contracts and are currently testing and validating the idea. Current users may also do validation, we'll apply smart-contract-based technical validation in this case. Our accreditation contributes to the blockchain's potential, we created a primary smart contract on the Ethereum network to put our idea to the test, this is a snapshot of the smart contract's design and implementation. Write some unit tests to confirm that methods return the right values and that state variables are populated correctly. Create integration tests to investigate the connections between the various contracts. As a backup to these other tactics, inheritance and dependency injection assist in ensuring that the desired behaviours are carried out exactly as planned.

## 4. Supply Chain Management in the Future

The ability to trace the origin of an item improves supply chain transparency, the blockchain documents a product's provenance, including the date, location, and quality. Consumers will be more confident in their purchases, and manufacturers will be at ease. Smart contracts may also be used to construct and store digital identities for parties in the supply chain. This method enables parties to verify the credentials of other parties easily, blockchain may also be used to control reputations. A smart contract can track inventories from the point of origin to the point of consumption, enhancing supply chain traceability. These intelligent sensors also provide location and environmental information (especially for perishable goods). The real-time product data aid decision-making rather than waiting for the problematic batch to arrive, it is better to activate a reserved batch of products in this case. The supply chain is adaptable and avoids bottlenecks.

Natural disasters, industrial strikes, and shipping concerns will all be handled efficiently. In the face of increased product competition, supply consistency may benefit a brand's consumer image. Smart contracts have the potential to improve supply chain operational and financial efficiency. Smart contracts on the distributed ledger manage multi-party supply chains and improve process efficiency. Saving money increases efficiency. Contractual agreements need less physical paperwork from the purchasing, accounting, and legal departments since they use trusted computer code. The removal of physical documents decreases labor.

Consumer-to-provider solutions offer a public ledger via which many individuals may access digital data about items, people, and events. Supply chain management using blockchain technology may help to overcome system management issues. The supply chain must evolve to meet changing customer needs. Supply chain standardization may assist marketing. Other than serial numbers and IDs, an RFID receiver may provide data. As commodities move through warehouses and transportation, the system automatically monitors shipments and stock whereabouts. RFID technology may be used in these systems to evaluate product quality and correct flaws. Product data may be tracked via collaboration or IoT throughout the shipping and storage processes. RFID-enabled supply chain networks can identify and penalize theft and other illicit activities in real-time. The manufacturer collects product data and embeds a QR code. The items are subsequently delivered to the distributor, who is notified. The new product predicts sales using machine intelligence and includes a consumer mobile app. This item is for sale. Product information is consistent. A communication platform is made up of websites and mobile applications. Blockchain technology becomes operational as soon as the genesis block is produced by scanning the QR code, you may learn about the product's origin, age, length, and expiry date.

This research suggests an illustrated new tracking paradigm, a blockchain smart contract for tracking agricultural supply chains. As a result, the conventional blockchain supply chain has been enhanced. It consists of four layers. All the first-layer activities, such as material procurement and sales, are managed by the producer agent. The products in the next layer are sorted, packaged, and processed by processor agents. Transport agents oversee all transportation throughout supplier networks. In this example, the retailing agent buys a product from the processing agency. Using decentralized blockchain smart contracts to create a unified supply chain means that the blockchain network can record every transaction. It is possible to validate the origin and processing, massive agricultural expansion is possible because of a revolutionary supply chain model. Clients may use the blockchain to track their orders, this strategy builds client trust, which leads to more sales.

## 5. Conclusion

Using blockchain, you may create a frictionless environment, it is, however, challenging to instil trust between farmers and purchasers. Because of current IoT-based agricultural systems, there is a lack of direct contact between farmers and market consumers. We combined IoT and blockchain for the food supply chain, and we devised an energy-efficient routing approach to extend the system's life. In the future smart agriculture and food supply chain paradigm, farmers will be trained on new crop data. The insect infestation, agricultural production, soil temperature, and soil quality will be measured via the Internet of Things. Crop monitoring allows for accurate crop tracking. Blockchain technology makes decentralized information networks safer, more accessible, and more enjoyable. With a smart model, the food supply chain will be more efficient and trustworthy. Blockchain technology makes supply chain management more efficient and transparent. We provide cutting-edge blockchain technology to optimize traditional supply networks. Because smart contracts eliminate the need for intermediaries, multi-agent systems manage the whole supply chain. Any supply chain may be secured and optimized by our automated system. We are safeguarding agriculture by using blockchain technology. This approach can verify product authenticity, track freight transit, and record transactions.

The study's agents also ensure that both parties adhere to the smart contract guidelines. If the agent discovers that a participant has not met the terms, they are punished. While monitoring and confirming orders, enhance the model's dependability and efficiency. We created an Ethereum smart contract in Solidity to put our hypothesis to the test. Researchers may utilize a hyper ledger fabric composer or multi-chain tools to test this proof of concept or model on a permissioned blockchain. It aims to solve two critical scientific problems. Examining existing supply chain issues and investigating how blockchain technology might assist in addressing them is a good start. The benefits of blockchain integration with supply networks are the subject of a well-researched and published paper on the issue. Ethereum's blockchain has an interplanetary file system and a proof of authority consensus mechanism. Payments may be handled directly by smart contracts, which improves performance. View the proposed smart contract paradigm, entity-relationship diagrams, and case studies. The immutability of ledger technology may increase supply chain security and trust, this method may be used for a variety of supply networks. Food data may be monitored, secured, and decentralised using blockchain technology, allowing for more transparency. The immutability of the data stored by a blockchain is one of its distinguishing features and a critical advantage for consumers. Everyone who is a part of the network has access to the specifications of every transaction that has occurred on the network.

## Figures and Tables

**Figure 1:** Displays a data-driven smart farm management cycle.

**Figure 2:** Food and agriculture supply chain process [7].

**Figure 3:** Blockchain technology in supply chain.

**Figure 4:** IoT and blockchain smart model.

**Figure 5:** Blockchain-based food supply chain.

**Figure 6:** IoT-based agriculture cluster farm and data transmission.

**Figure 7:** Network stability period and network life of proposed method and traditional IoT-based agriculture protocol.

## Data Availability

No data were used to support the findings of the study.
